The article "Expression EEG Multimodal Emotion Recognition Method Based on the Bidirectional LSTM and Attention Mechanism" was published in 2021. Journal: Comput Math Methods Med.

# Expression EEG Multimodal Emotion Recognition Method Based on the Bidirectional LSTM and Attention Mechanism

**DOI:** 10.1155/2021/9967592

**Published:** 2021-05-11

**Authors:** Yifeng Zhao, Deyun Chen

**Affiliations:** School of Computer Science and Technology, Harbin University of Science and Technology, Harbin, Heilongjiang 150080, China

## Abstract

Due to the complexity of human emotions, there are some similarities between different emotion features. The existing emotion recognition method has the problems of difficulty of character extraction and low accuracy, so the bidirectional LSTM and attention mechanism based on the expression EEG multimodal emotion recognition method are proposed. Firstly, facial expression features are extracted based on the bilinear convolution network (BCN), and EEG signals are transformed into three groups of frequency band image sequences, and BCN is used to fuse the image features to obtain the multimodal emotion features of expression EEG. Then, through the LSTM with the attention mechanism, important data is extracted in the process of timing modeling, which effectively avoids the randomness or blindness of sampling methods. Finally, a feature fusion network with a three-layer bidirectional LSTM structure is designed to fuse the expression and EEG features, which is helpful to improve the accuracy of emotion recognition. On the MAHNOB-HCI and DEAP datasets, the proposed method is tested based on the MATLAB simulation platform. Experimental results show that the attention mechanism can enhance the visual effect of the image, and compared with other methods, the proposed method can extract emotion features from expressions and EEG signals more effectively, and the accuracy of emotion recognition is higher.

## 1. Introduction

With the rapid development of computer and artificial intelligence technology, computer intelligence is paid more and more attention. Emotion recognition is one of the important research issues of human-computer interaction and the key technology of computer intelligence [1]. The purpose of emotion recognition research is to build a robot system that can recognize human emotions and give correct feedback so as to make the human-computer interaction process more friendly [2]. Emotion recognition is the detection of human emotional states by computer technology such as classification recognition; that is, humans hope to make computers feel, understand, and even express their own emotions very well through intelligent technology and, at the same time, hope to complete relevant instructions through human emotional manipulation computers and realize the computer intelligence of emotion calculation [3].

The commonly used emotional signals at present include external intuitive emotional signals such as voice and posture and internal bioelectrical signals such as electroencephalogram and electrocardiogram [4]. Among them, the voice signal is the most convenient and direct way to get each other's emotional state from many external emotional signals [5]. But for the speech process, deliberately concealed information cannot make an accurate judgment. For the intrinsic bioelectric signals such as EEG and ECG, although there is no intuitive expression of emotional information such as voice signals, the emotion recognition system built by bioelectric signals is more reliable because the bioelectric signals are not easy to be modified by subjective manipulation. Among the many bioelectrical signals, the EEG can reflect the activity of hundreds of millions of neurons in the cerebral cortex and has the characteristics of convenient collection, simple cost, and high time resolution [6]. Studies have shown that different emotional states reflect different EEG signals in the cortex of the brain. Therefore, EEG signals can be used as effective intrinsic bioelectrical signals to express human emotional information [7]. How to effectively process the EEG signal and extract the emotional information contained in the EEG signal is currently the main research issue of the emotion recognition of the EEG signal.

In order to build an emotion recognition system that is more in line with the human emotional processing mechanism, breaking through the bottleneck of multimodal emotion recognition technology which combines different physiological signals to assess emotional states has become a research hotspot [8]. The multimodal emotion recognition system can combine multimodal information and reduce the redundancy between different modes to make the emotional information complementary to each other so as to achieve a better emotion recognition effect [9]. Although some progress has been made in multimodal affective recognition technology, the current effect of affective recognition has not reached an ideal state due to the short research period. Therefore, how to construct a multimodal affective recognition system will be another key issue in affective computing research [10].

Based on the above analysis, an expression electroencephalogram multimodal affective recognition method based on the bidirectional LSTM and attention mechanism is proposed to solve the problems of the single mode, which are difficulty of deeply extracting signal characteristics and low accuracy of affective recognition.

1. The bilinear convolution network (BCN) has designed a new projection layer and uses a one-dimensional filter to extract the optimal feature space. Therefore, the proposed strategy based on BCN extracts facial expression features, converts the EEG signal into three bands of image sequences, and uses BCN to fuse its image features to obtain more accurate expression EEG multimodal affective features
2. In order to avoid the randomness or blindness of sampling methods, the attention mechanism is introduced in the LSTM network, and a characteristic fusion network with a three-layer bidirectional LSTM structure is designed to combine emoticons and EEG characteristics to improve the accuracy of emotion recognition

## 2. Related Works

Emotion is the role of the human cognitive process and conscious process, and it is an indispensable part of the human physiological process. Speech emotion recognition is relatively mature at present, and speech emotion recognition has been applied in different industries. The construction of a speech emotion recognition system mainly includes three parts: the establishment of a database, the extraction of emotion features, and the construction of an emotion classification model. In order to evaluate emotions more effectively, the research of the speech recognition system has been widely used by relevant researchers [11]. The establishment of an effective database is the basis of building a speech affective recognition system. Obtaining a subset of affective features that effectively represent the degree of emotional difference is the key to building a speech affective recognition system. The construction of a speech affective classification model is the key to achieving speech affective recognition. Reference [12] identifies three basic elements of the database, feature extraction, and classification method in the voice emotion recognition system, discusses the performance of the voice emotion recognition system, and uses the HMM (hidden Markov model), GMM (Gaussian mix model), and SVM (support vector machine) to achieve emotion recognition. A speech emotion recognition algorithm based on an improved stack kernel sparse depth model is proposed in Reference [13]. The algorithm is improved based on an automatic encoder, denoising automatic encoder, and sparse automatic encoder. The evaluation results on the test dataset show that the algorithm is better than the existing new algorithm in speech emotion recognition accuracy, but it is easy to be affected by the external environment in practical application, and there are many restrictions.

Among many bioelectrical signals, the EEG signal, as the product of brain neural activity, is more used in emotion recognition than other bioelectrical signals [14]. EEG signals are obtained by recording the potential changes in the cerebral cortex, which can be affected by external stimuli or human emotions, consciousness, and other activities. Reference [15] uses a classifier model to identify human emotional states or emotions through EEG signals and uses a classifier based on DBN (deep belief network) to classify and identify emotions using extracted features. Finally, the feasibility of the proposed method is analyzed from the indicators of accuracy, sensitivity, and specificity, and the results show that the proposed method can accurately identify emotions. Reference [16] provides an effective method of emotion recognition based on FAWT (flexible analytic wavelet transform). FAWT decomposes the EEG signal into different subband signals, uses the information potential to extract the features from the decomposition subband signal of the brain electrical signal, and then enters it smoothly into the random forest and support vector machine classifier that classifies the emotion. Compared with the existing method, the method shows better performance in human emotion classification. In the emotion recognition of electro-electrical signals, the current research difficulties are the establishment of effective databases and the extraction of EEG emotional characteristics; the above methods are based on a single modal database; although it has better popularity, the accuracy is not high.

At present, emotion recognition through a single signal has achieved a good recognition effect, but emotion recognition through a single signal is often disturbed by other signals, making the emotion recognition system in the process of emotion recognition have certain limitations. Therefore, in order to overcome the problem of the low recognition rate of the single modal emotional signal and the mutual influence between emotional signals, multimodal emotion recognition has become a research hotspot in emotion computing [17]. Multimodality is the combination of a variety of emotional signals, and various emotional signals complement each other. From the perspective of human perception of the emotional mechanism and processing mode, multimodal emotion recognition can more truly realize the simulation and reconstruction of a human emotional processing mechanism. So, the construction of a multimodal emotion recognition system is of great significance for the realization of emotion computing [18]. Reference [19] proposes a multimodal emotion recognition method that integrates speech and brain electrical signals, induces joy, sadness, anger, and neutral emotion through sound stimulation, collects the corresponding speech and brain electrical signals, extracts the nonlinear geometric and attribute characteristics of brainpower, constructs the characteristic fusion algorithm based on the constraint Boltzmann machine, and constructs the multimodal emotion recognition system by using the secondary decision algorithm through decision fusion. The results showed that the overall recognition rate of the multimodal emotion recognition system constructed by feature fusion was 1.08% and 2.75% higher than the single modal voice signal and brain electrical signal, respectively. However, the proposed method cannot quickly locate the emotional key information from the multimodal signals containing a large amount of redundant information, so the overall efficiency of the model needs to be improved. In Reference [20], a novel visual expression feature extraction and classification method based on the displacement of specific continuous landmarks in the continuous frame of voice is proposed. The discrete wavelet transform is used to analyze the displacement signal of the landmark, and a variety of dimensionality reduction schemes are used to reduce the complexity of the derived model and improve the efficiency. The experimental results on the SAVEE, RML, and eNTERFACE05 databases show the effectiveness of the proposed method of visual feature extraction, but the improvement of the interactive collaborative fusion of heterogeneous multimodal signals of human emotion can further improve the accuracy of recognition. The basic idea of the traditional multimodal emotion recognition method is to manually design and extract the features of each mode, then fuse the multimodal signals, and finally train the pattern classifier using the marked dataset. However, this kind of method has low efficiency in processing large-scale human emotion data [21]. In recent years, popular deep learning methods have a strong ability of feature expression.

At present, most of the emotion recognition methods based on EEG and face videos regard the signals of two modes as time series and construct the LSTM emotion recognition model for the two modes, respectively, to learn the recognition results of each sequence and finally fuse the recognition results at the decision level. Reference [22] established a psychophysiological database, which classified the EEG, GSR, and heart rate of 30 participants exposed to the affective virtual environment. 743 features were extracted from physiological signals. Then, by using feature selection techniques, the dimensions of the feature space are reduced to a smaller subset of only 30 features. Using KNN, SVM, distinguished analysis (DA), and classification tree (four classification techniques), the emotional psychophysiological database is classified into four emotional clusters and eight emotional tags. The experimental results show that physiological signals can be used to classify emotional experiences with high accuracy.

Although more and more researchers pay attention to multimodal emotion recognition technology, the overall emotion recognition rate is relatively low, which is not enough to be applied in real life. Therefore, multimodal emotion recognition will be the key research part in emotion computing [23, 24].

## 3. Feature Extraction Based on the Bilinear Convolution Network

The input signals for emotion recognition are facial expressions and electroencephalogram signals collected by the participants when they watch the emotion-induced video. Among them, the facial expression is the facial activity signal collected by the ordinary camera and belongs to the visual signal [25]. The EEG (electroencephalogram) signal refers to the electrophysiological signal generated by the spontaneous and rhythmic movement of brain neurons recorded in the scalp surface in chronological order, and it belongs to the physiological signal. EEG signals are collected by allowing participants to wear electrode brain caps while watching emotion-induced videos to obtain EEG signals from 32 different locations in the human cerebral cortex. It is difficult to fuse two heterogeneous signals directly so that the method proposed in this paper extracts the features with strong expression and generalization capabilities, while effectively interacting and synergizing the features of the two modes. The feature extraction process is shown in Figure 1.

For facial expressions, BCN is used to extract facial expression features. Compared with traditional feature extraction methods, BCN has a stronger ability to mine potentially distributed expression features of the data [26]. As shown in Figure 1, for EEG signals, the first step is to convert the EEG signals into image sequences of three bands. This kind of visualization processing preserves the time-space characteristics of the EEG signals while unifying the two modes into images. Then, the features of EEG images are extracted based on the BCN and spatial band attention mechanism, explained as follows:

*(1) Feature Extraction Process of the Facial Expression*. First, use the Faster RCNN model to detect the face area in the video frame, then use BCN to extract features from the face area, and finally use the full connection layer to process features to output the final feature vector *f*_*υ*,*n*_.

*(2) Feature Extraction Process of the EEG Signal*. First, the original EEG signal is removed by the wavelet soft threshold algorithm to get a relatively pure signal. Then, the EEG signal is divided into each segment with a duration of *T* (1/*T* corresponds to the frame rate of the facial expression) using the data processing method. At the same time, the spectrum energy information of *α*, *β*, and *θ* bands of EEG was extracted from the *t*-th band data, and the EEG images of three bands were visualized on the corresponding 32 electrodes of the electrode cap. As human emotional activation increases, *β*-wave forehead development increases significantly. Finally, BCN is used to extract layer features *f*_*α*,*n*_, *f*_*β*,*n*_, and *f*_*θ*,*n*_ from three bands of EEG images; then, the importance *f*_*n*_′ of the three groups of features is calculated using the spatial band attention mechanism, and the *f*_*n*_′ output eigenvector *x*_*e*,*n*_ is processed using the full connection layer. *f*_*n*_′ is calculated as

(1) $$\begin{array}{c} f_{n}^{\prime }=f_{\alpha ,n}\theta_{en,1}+f_{\beta ,n}\theta_{en,2}+f_{\theta ,n}\theta_{en,3}, \end{array}$$

where *θ*_*en*,1_, *θ*_*en*,2_, and *θ*_*en*,3_ represent the importance assigned to *f*_*α*,*n*_, *f*_*β*,*n*_, and *f*_*θ*,*n*_, respectively. The importance of each feature *θ*_*en*,*i*_ is as follows:

(2) $$\begin{array}{c} \theta_{en,i}=\frac{\exp\left(\omega_{h,i}h_{n-1}+b_{n,i}\right)}{\sum_{j=1}^{3}\exp\left(\omega_{h,j}h_{n-1}+b_{n,j}\right)},\;i=1,2,3, \end{array}$$

where *ω*_*h*,*i*_ is the weight matrix to be learned, *b*_*n*,*i*_ is the deviation, and *h*_*n*−1_ is the hidden state of *n* − 1 in the multilayer network.

The network structure of BCN is shown in Figure 2, which consists mainly of six network layers, namely, two projection layers, one one-dimensional convolution layer, two full connection layers, and one Softmax layer. BCN and traditional CNN have a big difference, mainly reflected in its network input as the SIFT feature matrix rather than the original picture, and we designed a new projection layer to find the optimal combination between key points and the optimal feature space and the characteristic direction of the use of the one-dimensional filter to learn the characteristics with high differentiation [27].

When constructing the input feature matrix, assuming that *M* key points have been located from each expression image and the *N*-dimensional SIFT feature vector is extracted for each key point, then the input of BCN is an *M* × *N* feature matrix. The feature matrix is then entered into the BCN for feature learning and classification [28]. In this process, the eigenmatrix first passes through a projection layer containing the multichannel left multiple projection matrix to find the optimal combination of key points. Similarly, in the second projection layer, the right multiple projection matrix will further optimize the feature space.

Suppose *H*_*t*_ = {*h*_*t*,*j*_^(l)^|*j* = 1, ⋯, *C*_*l*_}(*t* = 1, ⋯, *N*_*l*_) is the *t*-th left multiple projection matrix containing *C*_l_ channels, *h*_*t*,*j*_^(l)^ is the *j*-th channel of *H*_*t*_, and *N*_l_ is the number of left multiple projection matrices; then, the left multiple projection layer can be defined as

(3) $$\begin{array}{c} O_{t}=\overset{C_{\text{l}}}{\underset{j=1}{\sum }}h_{t,j}^{\left(\text{l}\right)}I_{j},\;t=1,2,\cdots ,N_{\text{l}}, \end{array}$$

where *O*_*t*_ is the *t* channel of the output feature and *I*_*j*_ is the *j* channel of the input matrix. Similarly, for the projection layer of the right multiple projection matrix, we have

(4) $$\begin{array}{c} O_{t}=\overset{C_{\text{r}}}{\underset{j=1}{\sum }}h_{t,j}^{\left(\text{r}\right)}I_{j},\;t=1,2,\cdots ,N_{\text{r}}. \end{array}$$

After the above operation, the right multiple projection layer projects each row of the input matrix from the current feature space to another feature space with a strong character and also plays the role of feature dimension reduction.

A one-dimensional convolution layer uses a set of multichannel filters to filter the characteristics entered, and the layer is often used in conjunction with the maximum pooling layer. In the process of convolution of input features, the one-dimensional filter can produce a strong response to local features with a specific structure and suppress the response value of local features different from the structure, which makes the filter capture the key local structure in the feature matrix. After the filtering operation, the convolution response is maximized to obtain the output characteristics of the convolution layer.

The output of the maximum pooling layer will pass through a nonlinear activation function to increase the flexibility of BCN before it is transferred into the full connection layer. Assuming that the output matrix of the maximum pooling layer can be represented by *Q* = [*Q*_*c*,*i*,*j*_]_*C*×*I*×*J*_ (where *C*, *I*, and *J* represent the number of channels, the number of rows, and the number of columns of the matrix, respectively), the nonlinear activation process can be expressed as follows:

(5) $$\begin{array}{c} F_{c,i,j}=\tanh\left(b_{c}+Q_{c,i,j}\right). \end{array}$$

In the formula, *F* = [*F*_*c*,*i*,*j*_]_*C*×*I*×*J*_ is the output matrix of the nonlinear response function, and the size of the matrix is the same as that of the input matrix, and *B* is the element value in row D and column E on the *c*-th channel of the matrix.

In the formula, *F* = [*F*_*c*,*i*,*j*_]_*C*×*I*×*J*_ represents the output matrix of the nonlinear response function, and the size of the matrix is the same as that of the input matrix, and *F*_*c*,*i*,*j*_ represents the element value on the *c* channel of the matrix *F* that is in column *j* and row *i*. The nonlinear activation function is a hyperbolic tangent function, which is represented by tanh(·), while *b*_*c*_ represents the global offset to the *c* channel of the input matrix during the nonlinear transformation.

The full connection layer and Softmax layer used in the BCN are the same as those in traditional CNN, where the full connection layer first stretches the nonlinear transformation-after response matrix to vectors and projects it, then finally classifies it through the Softmax layer. When training BCN, the training dataset is first divided into several batches of data and then input into the network in turn. According to the defined loss function, the difference between the prediction probability and the actual category of samples is calculated.

## 4. Interactive Collaborative Process Based on the Bidirectional LSTM and Attention Mechanism

### 4.1. Feature Fusion

Feature fusion is used to integrate different types of features to achieve redundancy and get features that are conducive to analysis and processing. Generally, there are two intuitive fusion methods in neural networks: add and concatenate. The add method is the addition of feature maps, which increases the amount of information describing the features of the image, but the dimension describing the image itself does not increase, but the amount of information in each dimension is increasing, which is obviously beneficial for the final image classification. Concatenate is a merge of the number of channels; that is, the features describing the image itself increase, while the information under each feature does not increase. Direct stitching of multilayered information in the network cannot make better use of the complementarity between features, so consider mapping features to multiple subspaces for weighted fusion and stitching them together.

Similar to the general neural network method, the number of subspaces is a superparameter. For each subspace, the corresponding central variables are defined and randomly initialized, and the mapping matrix is also initialized at the same randomness, calculating the adaptive weight based on the distance between the feature and the central variable. As with neural network model parameters, eventually, all mapping matrices and central variables are obtained by training neural networks through BP algorithms.

Assuming that layer *n* features are extracted, each feature is represented by *f*_*i*_(*i* = 1, 2, ⋯, *n*), the feature dimension is *df*, the mapping matrix SW = [SW_1_, SW_2_, ⋯, SW_*k*_] ∈ *R*^*df*×*dk*^ is defined, the features are mapped to a subspace, weighted fusion is performed under the subspace, and the central variable *M* = [*M*_1_, *M*_2_, ⋯, *M*_*k*_] ∈ *R*^*t*×*dk*^ is defined, where *df* = *k* × *dk* and *k* represent the number of subspaces set, and *dk* represent the feature dimension mapped to a subspace. The adaptive weights are computed, and the subspace features are stitched together. The feature fusion process is as follows:

(6) $$\begin{array}{c} {\text{sw}}_{i,j}=e^{-\left(1/df\right){\left\|F_{i}{\text{SW}}_{j}-M_{j}\right\|}_{2}^{2}},\\ {\text{Sf}}_{j}=\overset{n}{\underset{i=1}{\sum }}{\text{sw}}_{i,j}\left(f_{i}{\text{SW}}_{j}\right),\\ \text{SF}=\text{Concat}\left({\text{Sf}}_{1},{\text{Sf}}_{2},\cdots ,{\text{Sf}}_{k}\right). \end{array}$$

In the formula, sw_*i*,*j*_ represents the weight corresponding to the *i* feature in the *j* subspace, Sf_*j*_ represents the feature after the *j* subspace is added and fused by weight, and SF indicates the final feature fusion formed by the stitching of each subspace feature fusion.

### 4.2. LSTM with the Attention Model

The attention model contains two kinds of attention mechanisms. The calculation process of the soft attention mechanism is subtle, can be easily embedded in a known framework, and can spread the gradient in the attention model [29]. The hard attention mechanism is a random process in which the hidden state is sampled with a certain probability. In order to transfer the gradient, Monte Carlo sampling is usually used to estimate the gradient, which makes the hard attention mechanism not well embedded as a module in known models. Therefore, in order to facilitate model training, the soft attention mechanism is introduced into the LSTM network to form the AM-LSTM (attention mechanism-LSTM) network.

The attention model weights the input vector *x*_*t*_ in each time step to generate a new vector *a*_*t*_ as follows:

(7) $$\begin{array}{c} a_{t}=\varphi \left(\omega_{xa}x_{t}+\omega_{xa}h_{t-1}+b_{a}\right). \end{array}$$

In the formula, *φ* represents the sigmoid activation function, *ω* represents the weight matrix, and *b*_*a*_ represents the offset vector. The importance of each element in the input vector *x*_*t*_ is determined by the current input *x*_*t*_ and hidden state *h*_*t*−1_.

The attention response is multiplied by the point of the input vector to output a new input vector ${\overset{⌢}{x}}_{t}$, which is calculated as follows:

(8) $$\begin{array}{c} {\overset{⌢}{x}}_{t}=a_{t}⊗x_{t}. \end{array}$$

The activation function in the LSTM network module then iteratively calculates based on the new input vector element. The computational unit of the recurrent neural network for the attention module is formalized as follows:

(9) $$\begin{array}{c} i_{t}=\sigma \left(\omega_{xi}{\overset{⌢}{x}}_{t}+\omega_{hi}h_{t-1}+b_{i}\right),\\ f_{t}=\sigma \left(\omega_{xf}{\overset{⌢}{x}}_{t}+\omega_{hf}h_{t-1}+b_{f}\right),\\ o_{t}=\sigma \left(\omega_{xo}{\overset{⌢}{x}}_{t}+\omega_{ho}h_{t-1}+b_{o}\right),\\ c_{t}=f_{t}\times c_{t-1}+i_{t}⊗\Phi \left(\omega_{xc}{\overset{⌢}{x}}_{t}+\omega_{hc}h_{t-1}+b_{c}\right),\\ h_{t}=o_{t}⊗\tanh\left(c_{t}\circ f_{p}\right). \end{array}$$

*i*, *f*, *o*, and *c* are the input gate, forget gate, output gates, and memory units. To prevent overfitting, the dropout algorithm is introduced in the training process. In the training process, the parameter of the weight layer is randomly sampled with a certain probability *p*, and *f*_*p*_ is the vector produced by the Bernoulli distribution with probability *p*. Most attention mechanisms use Softmax to calculate the weights of each element so that the sum of weights is guaranteed to be 1, but in this case, the attention weights between elements influence each other, even if they are of the same importance. So using the sigmoid activation function, the weights can be normalized between 0 and 1.

### 4.3. Feature Fusion Based on the Bidirectional Long-Term and Short-Term Memory Network

Feature fusion can be divided into early fusion and delayed fusion. Early fusion cannot learn the time series dynamics of each feature for tasks that require time series modeling. Delayed fusion may lose the time series information that exists in the feature representation of multiple models. To solve the above problem, the proposed method designs a three-layer bidirectional LSTM network to fuse features, as shown in Figure 3.

The first layer of the bidirectional LSTM network uses a separate bidirectional LSTM layer to model each feature in time series. The second layer combines hidden features from the RGB image model and hidden features from the depth image model using linear functions, using the sigmoid function to add nonlinear factors, and generating new feature representations at each time step. The third layer uses the bidirectional LSTM network to model the output of the second layer in time series.

Assuming that *x*_*t*_^*m*^ is the feature representation extracted from RGB or depth models at time *t*, the three levels of the network are described as follows:

*(1) Layer 1*. The input of this layer is *x*_*t*_^*m*^, assuming that Ψ represents a two-way long-term and short-term memory network layer, and *h*_*t*_^*m*^ is the implicit layer representation of *t* moment.

(10) $$\begin{array}{c} h_{t}^{m}=\Psi \left(x_{t}^{m}\right). \end{array}$$

*(2) Layer 2*. This layer uses a linear function to fuse the characteristics of the hidden layer and a sigmoid function to add nonlinear factors.

(11) $$\begin{array}{c} f_{t}=\sigma \left(\omega \left(h_{t}^{\text{RGB}},h_{t}^{\text{BCN}}\right)+b\right). \end{array}$$

In the formula, *ω* is the weight matrix, *h*_*t*_^RGB^ is the hidden layer of the RGB feature at time *t*, *h*_*t*_^BCN^ is the hidden layer of the BCN feature, *b* is the offset, and *σ* is the sigmoid function.

*(3) Layer 3*. This layer uses a bidirectional LSTM layer to model the time series of fused feature *f*_*t*_.

(12) $$\begin{array}{c} h_{t}^{f}=\Psi \left(f_{t}\right). \end{array}$$

The final output is used as the input to the fully connected layer for final prediction.

### 4.4. Loss Function Used in Training

The BP (backpropagation) algorithm is commonly used in training neural networks, and the most intuitive function of the loss function is to update the model parameters by calculating its backpropagation gradient. The use of different loss functions tends to make the model more focused on learning some aspects of the data characteristics and can better guarantee the unique characteristics of the extracted features later, so the loss function has a guiding effect in network optimization [30].

Classification networks are generally trained with the cross-entropy loss function, which is as follows:

(13) $$\begin{array}{c} L_{S}=-\frac{1}{N}\overset{N}{\underset{i=1}{\sum }}\log\frac{e^{\omega_{yi}^{T}x_{i}+b_{yi}}}{\sum_{j=1}^{c}e^{\omega_{j}^{T}x_{i}+b_{j}}}, \end{array}$$

where *ω*_*j*_^*T*^*x*_*i*_ + *b* represents the full connection layer output and *yi* represents the real category label corresponding to the input sample. The essence of the loss function decline is to increase the proportion so that the samples of this class fall more within the decision boundary of this class.

However, for facial expression recognition, the cross-entropy loss function cannot guarantee that the distance between classes of extracted features increases. It mainly considers whether the samples can be classified correctly and lacks the constraint of the distance between classes and within classes [31]. Generally, the problem of the loss function in face recognition is solved in two ways. On the one hand, it combines the measure learning method; on the other hand, it is improved on the basis of this Softmax cross-entropy loss function. Add an additional loss function after the cross-entropy loss function to strengthen the constraint on the interclass distance, making the interclass feature distance of the same sample become compact but not sufficiently constrained between classes [32, 33]. The cross-entropy loss function is improved directly by normalizing *ω* and *x* and converting them to cosine distances.

(14) $$\begin{array}{c} L=-\frac{1}{N}\overset{N}{\underset{i=1}{\sum }}\log\frac{e^{\cos\theta_{yi}}}{\sum_{j=1}^{c}e^{\cos\theta_{j}}}. \end{array}$$

Then, introduce the interval constraint and use the AM-Softmax method to calculate the following:

(15) $$\begin{array}{c} L=-\frac{1}{N}\overset{N}{\underset{i=1}{\sum }}\log\frac{e^{\text{s}\left(\cos\theta_{yi}-m\right)}}{e^{\text{s}\left(\cos\theta_{yi}+m\right)}+\sum_{j=1,j\neq yi}^{c}e^{\text{s}\cos\theta_{j}}}. \end{array}$$

For all features, feed into the Softmax classifier, using the above loss function, as follows:

(16) $$\begin{array}{c} \text{loss}\left(F\right)=\overset{n}{\underset{i=1}{\sum }}L\left(f_{i}\right). \end{array}$$

On this basis, the loss of the fused part is added, and the loss function calculation process is shown in Figure 4.

For the feature fusion part, the fused features are fed into the Softmax classifier, and loss(SF) is used to represent the above loss function. For the decision fusion section, loss(DF) is used to represent the above loss function [34, 35]. Add all the loss functions as the final loss function, in the following form:

(17) $$\begin{array}{c} \text{Loss}=\text{loss}\left(F\right)+\text{loss}\left(\text{SF}\right)+\text{loss}\left(\text{DF}\right). \end{array}$$

## 5. Experimental Scheme and Result Discussion

To verify the validity of the proposed method, the MATLAB simulation platform experimented on the MAHNOB-HCI dataset and the DEAP dataset and used RA (recognition accuracy) and F1-score as evaluation indicators for recognition. In addition, the two-dimensional arousal-valence emotional space is used in the experiment, and its principle is shown in Figure 5.

In the figure, the horizontal valence represents the validity, indicating the positive and negative degrees of emotion, and the vertical arousal represents the activation degree, indicating the intensity and depression of emotion. By setting validity and wakefulness, complex and subtle emotions can be expressed and distinguished, such as ecstasy and cheerfulness, which describe varying degrees of pleasure and elation, which express two different kinds of joy. The two-dimensional affective space has become the main dimensional space used for dimension affective recognition because of its simple structure and rich emotional expression ability.

The MAHNOB-HCI dataset is a multimodal affective recognition and latent labeling dataset, which includes 527 sets of original face videos and audio and electroencephalogram signals collected from 27 participants who watched 20 videos. After watching each video, the participants used the activation and effect value of the calibration emotions, which were divided into 9 levels (1-9, respectively). Emotions are also calibrated using discrete affective tags, which categorized the activation and validity of experimenters' emotions into three categories.

DEAP is a multimodal emotion recognition dataset that includes face videos, external physiological signals, and electroencephalogram signals collected from 32 participants during 40 music videos. The data of 10 participants do not include facial expression videos. After viewing each video, the participants used the activation and validity of the calibrated emotions (values 1-9). The dataset divides emotional activation and validity into three levels according to their numerical size.

The results of model recognition are evaluated using two indicators: recognition accuracy and F1-score, where recognition accuracy RA represents the percentage of the number of samples correctly classified in the test set to the total number of samples in the test set. F1-score is a statistical measure of the accuracy of a multiclassification model. It can be viewed as a weighted average of model accuracy (precision) and recall rate (recall), which can take into account both the model accuracy and the recall rate. Recognition accuracy and F1-score are calculated as follows:

(18) $$\begin{array}{c} \text{RA}=\frac{N_{\text{TP}}}{N_{\text{data}}},\\ \text{F}1=\frac{2N_{\text{TP}}}{2N_{\text{TP}}+N_{\text{FP}}+N_{\text{FN}}}. \end{array}$$

In the formula, *N*_data_ represents the total number of samples of emotion data in the test set; *N*_TP_, *N*_FP_, and *N*_FN_ represent the total number of positive, false, and missed tests in all the test samples, respectively.

### 5.1. Visual Effect Comparison of the Attention Mechanism

Select samples from the MAHNOB-HCI dataset for a single set of emotion recognition tests and visualize the emotional key information on each step to Figures 6 and 7. Only four time steps are selected to visualize the time domain attention mechanism. The top bar in the graph represents the importance of three bands of EEG signals *α*, *β*, and *θ* at each time from bottom to top.

As you can see from the above two figures, the proposed method can locate valid information quickly and accurately and analyze the data more frequently in areas of valid information to obtain more accurate identification results. As can be seen from Figure 6, as the participants become more nervous (and more emotionally active), the EEG *β*-wave gradually dominates, which is consistent with the conclusion that the EEG *β*-wave in physiology dominates when humans are in an emotional state of stress, anxiety, panic, and so on. With the enhancement of the EEG *β*-wave, the human body will be more and more in a tense state. Under this condition, the human body and mind energy expenditure is rapid, and it is easy to feel pressure and fatigue. As can be seen from Figure 7, *α*-wave dominates when the human emotional state remains stable at a low activation level. Physiological studies have shown that when the main frequency of the human brain wave is *α*-wave, the human being is awake and relaxed, and it is also the best state for human thinking.

### 5.2. Comparison of the Learning Effect on Facial Emotion Significant Features

In the learning phase of facial expression features, four methods (proposed method and References [14, 20, 28]) were used to compare the results of feature learning based on the DEAP dataset in the two dimensions of arousal and valence, respectively, as shown in Figures 8 and 9. The *R*-squared coefficient and loss function Loss are used as the evaluation indicators of feature learning. The *R*-squared coefficient of the regression task represents the degree of fit between the predicted value and the label value by calculating the change of the data. The larger the value of the *R*-squared coefficient, the better the fit degree and the better the feature extraction effect. The *R*-squared coefficient function is as follows:

(19) $$\begin{array}{c} R^{2}=1-\frac{\sum {\left(Y_{\text{act}}-Y_{\text{pre}}\right)}^{2}}{\sum {\left(Y_{\text{act}}-\bar{Y}\right)}^{2}}. \end{array}$$

In the formula, *Y*_act_ is the emotional reality tag sequence, *Y*_pre_ is the emotional prediction value sequence, and $\bar{Y}$ is the average value of the emotional reality tag sequence.

From Figure 8, it can be seen that compared with other methods, the proposed method has the highest *R*-squared coefficient on the arousal dimension, and the loss is very low, which is close to 0.05, indicating that the feature extraction effect is the best. As can be seen from Figure 9, the squared coefficient of the proposed method is 0.63, the loss is very close to 0.002, and the network structure is simpler than several other methods. Therefore, the proposed method achieves better feature extraction results in the two-dimensional arousal-valence emotional state space.

### 5.3. Compared with the Dimensional Emotion Recognition Results of Other Methods

The two-dimensional emotional spatial expression was used to compare the results of dimensional affective recognition with those of References [16, 19, 20] in the MAHNOB-HCI dataset, as shown in Table 1.

As can be seen from Table 1, although the proposed method is inferior to the optimal method in terms of loss, the correlation coefficient better reflects the degree of fit between the emotional prediction value and the emotional tag value. Moreover, the recognition accuracy of the proposed method has exceeded the results of many methods, and the recognition accuracy of the hierarchical attention mechanism built on this basis performs best. Finally, the loss is optimized and the accuracy of the recognition rate is 0.749 and 0.706 in two dimensions, respectively, indicating that the proposed method can more effectively extract the emotional characteristics of the emoticon and the brain electrical signal to combine.

### 5.4. Comparison of Results from Multiple Emotion Recognition Methods

To demonstrate the performance of the proposed method, the results of this paper are compared with those of References [16, 19, 20], as shown in Table 2.

As can be seen from Table 2, the recognition accuracy and F1 of the proposed method are significantly improved compared with those of other methods. Because other methods directly analyze multimodal emotional signals that contain a lot of redundant information, the proposed method introduces the attention mechanism, which compresses the redundant information and improves the accuracy. On the MAHNOB-HCI dataset, the accuracy of affective activation recognition and F1 were improved by 1.1% and 0.021, respectively, and the accuracy of affective efficacy value recognition and F1 were improved by 0.4% and 0.024, respectively, compared with the methods in Reference [19], which showed better recognition results. And the recognition accuracy on the DEAP dataset is higher than that on the MAHNOB-HCI dataset because the DEAP dataset has more information, which is conducive to feature learning and classification.

In addition, it can be seen from Table 2 that the recognition of the emotional effect value is better than that of emotional activation. This is because the degree of emotional activation is used to show the degree of emotional motivation, and the value of the emotional effect is used to show whether people are good or bad in evaluating their emotional state. Compared with the value of the emotional effect, it is easier to analyze and understand intuitively. In particular, FAWT in Reference [16] decomposes EEG signals into different subband signals on the MANOB-HCI dataset, extracts features from them using the information potential, and smoothes them into random forests and SVM classifiers that classify emotions. It achieves good results in validity value recognition. Overall, the method proposed is more effective.

## 6. Conclusion

At present, most emotion recognition focuses on speech signals, facial expressions, ECG, EEG, and other bioelectrical signals. However, when the emotional signal of a single channel is interfered by other signals, the emotion recognition rate is often reduced. Therefore, a multimodal emotion recognition method based on the bidirectional LSTM and attention mechanism is proposed. Facial expression and EEG features are extracted based on BCN, and the attention mechanism is introduced into the LSTM network. Facial expression and EEG features are fused by a feature fusion network with a three-layer bidirectional LSTM structure to improve the accuracy of emotion recognition. The proposed method is tested on MAHNOB-HCI and DEAP datasets based on the MATLAB simulation platform. The experimental results show that the attention mechanism can enhance the visual effect of the image, and compared with other methods, the proposed method can extract emotion features in expressions and EEG signals more effectively and achieve a more accurate emotion recognition effect.

In real life, different emotions often have a certain correlation; for example, sad emotions often contain certain anger. Therefore, the emotion recognition system based on the relationship between emotions can reflect the human emotional information more effectively. So, the establishment of an effective emotion recognition model will be the focus of the next step of emotion recognition research.

## Figures and Tables

**Figure 1:** Feature extraction process of the facial expression and EEG signal.

**Figure 2:** Network structure of BCN.

**Figure 3:** Structure diagram of a three-layer bidirectional LSTM network.

**Figure 4:** Calculation process of the loss function.

**Figure 5:** Schematic diagram of the two-dimensional arousal-valence emotional state space.

**Figure 6:** Visualization results of the attention mechanism in high activation data samples.

**Figure 7:** Visualization results of the attention mechanism in low activation data samples.

**Figure 8:** Arousal dimension video emotion salient feature learning results.

**Figure 9:** Valence dimension video emotion salient feature learning results.

**Table 1:** Comparison of dimensional emotion recognition results of different methods.

	Arousal		Valence	
	*R* ^2^	Loss	*R* ^2^	Loss
Ref. [16]	0.442	0.263	0.477	0.174
Ref. [19]	0.535	0.181	0.469	0.115
Ref. [20]	0.687	0.152	0.642	0.338
The proposed method	0.749	0.174	0.706	0.127

**Table 2:** Comparison of recognition results of different methods.

	Arousal		Valence	
	RA (%)	F1	RA (%)	F1
Ref. [16]/MAHNOB-HCI	67.8	0.620	74.8	0.742
Ref. [19]/MAHNOB-HCI	73.5	0.711	74.9	0.715
Ref. [20]/MAHNOB-HCI	63.4	—	66.7	—
The proposed method/MAHNOB-HCI	74.6	0.732	75.3	0.739
The proposed method/DEAP	86.8	—	86.2	—

## Data Availability

The data included in this paper are available without any restriction.

## References

[1] Gabriels K. (2019). Response to uncertainty in emotion recognition. *Journal of Information Communication and Ethics in Society*.

[2] Singh L., Singh S., Aggarwal N. (2019). Improved TOPSIS method for peak frame selection in audio-video human emotion recognition. *Multimedia Tools and Applications*.

[3] Ozseven T. (2019). A novel feature selection method for speech emotion recognition. *Applied Acoustics*.

[4] Song P., Zheng W., Zhao L. (2018). Joint subspace learning and feature selection method for speech emotion recognition. *Qinghua Daxue Xuebao/Journal of Tsinghua University*.

[5] Li J., Qiu S., Shen Y.-Y., Liu C.-L., He H. (2020). Multisource transfer learning for cross-subject EEG emotion recognition. *IEEE Transactions on Cybernetics*.

[6] Liu Z. T., Xie Q., Wu M., Cao W. H., Mei Y., Mao J. W. (2018). Speech emotion recognition based on an improved brain emotion learning model. *Neurocomputing*.

[7] Hsu Y. L., Wang J. S., Chiang W. C., Hung C. H. (2020). Automatic ECG-based emotion recognition in music listening. *IEEE Transactions on Affective Computing*.

[8] Raheel A., Anwar S. M., Majid M. (2019). Emotion recognition in response to traditional and tactile enhanced multimedia using electroencephalography. *Multimedia Tools and Applications*.

[9] Dong Y., Yang X., Zhao X., Li J. (2019). Bidirectional convolutional recurrent sparse network (BCRSN): an efficient model for music emotion recognition. *IEEE Transactions on Multimedia*.

[10] Huang Y., Tian K., Wu A., Zhang G. (2019). Feature fusion methods research based on deep belief networks for speech emotion recognition under noise condition. *Journal of Ambient Intelligence and Humanized Computing*.

[11] Li Y., Zheng W., Cui Z., Zong Y., Ge S. (2019). EEG emotion recognition based on graph regularized sparse linear regression. *Neural Processing Letters*.

[12] Deepika C. (2020). Speech emotion recognition feature extraction and classification. *International Journal of Advanced Trends in Computer Science and Engineering*.

[13] Wei P., Zhao Y. (2019). A novel speech emotion recognition algorithm based on wavelet kernel sparse classifier in stacked deep auto-encoder model. *Personal and Ubiquitous Computing*.

[14] Zhang T., Zheng W., Cui Z., Zong Y., Li Y. (2019). Spatial–temporal recurrent neural network for emotion recognition. *IEEE Transactions on Cybernetics*.

[15] Wankhade S. B., Doye D. D. (2020). Deep learning of empirical mean curve decomposition-wavelet decomposed EEG signal for emotion recognition. *International Journal of Uncertainty, Fuzziness and Knowledge-Based Systems*.

[16] Gupta V., Chopda M. D., Pachori R. B. (2019). Cross-subject emotion recognition using flexible analytic wavelet transform from EEG signals. *IEEE Sensors Journal*.

[17] Jain N., Kumar S., Kumar A., Shamsolmoali P., Zareapoor M. (2018). Hybrid deep neural networks for face emotion recognition. *Pattern Recognition Letters*.

[18] Hwang S., Ki M., Hong K., Byun H. Subject-independent EEG-based emotion recognition using adversarial learning.

[19] Ma J., Sun Y., Zhang X. (2019). Multimodal emotion recognition for the fusion of speech and EEG signals. *Xi'an Dianzi Keji Daxue Xuebao/Journal of Xidian University*.

[20] Rahdari F., Rashedi E., Eftekhari M. (2019). A multimodal emotion recognition system using facial landmark analysis. *Iranian Journal of ence and Technology, Transactions of Electrical Engineering*.

[21] Zhang S., Zhang S., Huang T., Gao W., Tian Q. (2018). Learning affective features with a hybrid deep model for audio–visual emotion recognition. *IEEE Transactions on Circuits and Systems for Video Technology*.

[22] Moghimi M., Stone R., Rotshtein P. (2020). Affective recognition in dynamic and interactive virtual environments. *IEEE Transactions on Affective Computing*.

[23] Wasser C. I., Evans F., Kempnich C. (2018). Emotion recognition in Parkinson's disease: static and dynamic factors. *Neuropsychology*.

[24] Fang W. C., Wang K. Y., Fahier N., Ho Y. L., Huang Y. D. (2019). Development and validation of an EEG-based real-time emotion recognition system using edge AI computing platform with convolutional neural network system-on-chip design. *IEEE Journal on Emerging and Selected Topics in Circuits and Systems*.

[25] Wu C., Huang C., Chen H. (2018). Text-independent speech emotion recognition using frequency adaptive features. *Multimedia Tools & Applications*.

[26] Haritha C. V., Thulasidharan P. P. (2018). Multimodal emotion recognition using deep neural network- a survey. *INTERNATIONAL JOURNAL OF COMPUTER ENCES AND ENGINEERING*.

[27] Ye L., Wang P., Le Wang H. F., Seppänen T., Alasaarela E. (2018). A combined motion-audio school bullying detection algorithm. *International Journal of Pattern Recognition and Artificial Intelligence*.

[28] Saha A., Pradhan S. N. (2018). Facial expression recognition based on eigenspaces and principle component analysis. *International Journal of Computational Vision & Robotics*.

[29] Feng H., Golshan H. M., Mahoor M. H. (2018). A wavelet-based approach to emotion classification using EDA signals. *Expert Systems with Applications*.

[30] Pal R. (2018). Emotion recognition using facial expression. *International Journal on Computer ence & Engineering*.

[31] Nguyen H.-D., Yeom S., Lee G.-S., Yang H.-J., Na I.-S., Kim S.-H. (2019). Facial emotion recognition using an ensemble of multi-level convolutional neural networks. *International Journal of Pattern Recognition and Artificial Intelligence*.

[32] Athishmon F., Narayanan N., Suthendran K. (2018). Recognizing spontaneous emotion from the eye region under different head poses. *International Journal of Pure and Applied Mathematics*.

[33] Hu M., Wang H., Wang X., Yang J., Wang R. (2019). Video facial emotion recognition based on local enhanced motion history image and CNN-CTSLSTM networks. *Journal of Visual Communication & Image Representation*.

[34] Bo H., Ma L., Liu Q., Xu R., Li H. (2019). Music-evoked emotion recognition based on cognitive principles inspired EEG temporal and spectral features. *International Journal of Machine Learning and Cybernetics*.

[35] Yang Y., Wu Q. M. J., Zheng W. L., Lu B. L. (2018). EEG-based emotion recognition using hierarchical network with subnetwork nodes. *IEEE Transactions on Cognitive and Developmental Systems*.

